# A Semiautomated Deep Learning Approach for Pancreas Segmentation

**DOI:** 10.1155/2021/3284493

**Published:** 2021-07-02

**Authors:** Meixiang Huang, Chongfei Huang, Jing Yuan, Dexing Kong

**Affiliations:** ^1^The School of Mathematical Sciences, Zhejiang University, Hangzhou 310027, China; ^2^The School of Mathematics and Statistics, Xidian University, Xi'an 710069, China

## Abstract

Accurate pancreas segmentation from 3D CT volumes is important for pancreas diseases therapy. It is challenging to accurately delineate the pancreas due to the poor intensity contrast and intrinsic large variations in volume, shape, and location. In this paper, we propose a semiautomated deformable U-Net, i.e., DUNet for the pancreas segmentation. The key innovation of our proposed method is a deformable convolution module, which adaptively adds learned offsets to each sampling position of 2D convolutional kernel to enhance feature representation. Combining deformable convolution module with U-Net enables our DUNet to flexibly capture pancreatic features and improve the geometric modeling capability of U-Net. Moreover, a nonlinear Dice-based loss function is designed to tackle the class-imbalanced problem in the pancreas segmentation. Experimental results show that our proposed method outperforms all comparison methods on the same NIH dataset.

## 1. Introduction

Pancreatic diseases are relatively hidden and difficult to detect and cure, especially for pancreatic cancers, which have high mortality rate worldwide [1]. Accurate pancreas segmentation from 3D CT scans can provide assistance to doctors in the diagnosis of pancreas diseases, such as volumetric measurement and analysis for diabetic patients, as well as surgical guidance for clinicians [2]. However, it is challenging to segment the pancreas due to the large anatomical variability in pancreas position, size, and shape across patients (as shown in Figure 1). Moreover, the ambiguous boundaries around the pancreas with its adjacent structures further increase the difficulty of pancreas delineation.

Traditional methods on abdominal pancreas segmentation mainly have statistical shape models [3, 4] or multi-atlas techniques [5, 6]. Wolz et al. proposed a fully automated method based on a hierarchical atlas registration and weighting scheme for abdominal multiorgan segmentation [6]. This method was evaluated on a database of 150 CT scans and achieved Dice score of 70% for the pancreas. Karasawa et al. exploited the vasculature around the pancreas to better select atlases for pancreas segmentation [7]. This method was evaluated on 150 abdominal CT scans and obtained an average Dice score of 78.5%. However, the performance of atlas-based methods highly relies on the selection of atlases and the accuracy of the image registration algorithm. Above all, it is difficult to select atlases that are general enough to cover all variabilities in the pancreas across different patients.

Convolutional networks [8, 9] have achieved great success in medical image segmentation, which also boost the performance of pancreas segmentation. U-Net [10], a semantic segmentation architecture, attracted great attentions from researchers by exploiting multilevel feature fusion. The skip connections in U-Net are used to incorporate high-resolution low-level feature maps from the encoding branch into the decoding branch of U-Net to alleviate the important information loss caused by successive downsampling and then refine and recover target details. Namely, using skip connections to fuse multilevel feature tensors can effectively localize and segment target organs [11]. Many works [12–14] have demonstrated that U-Net is a good framework for semantic segmentation tasks, especially for small datasets. Since the pancreas is a small, soft organ in the abdomen, most pancreas segmentation algorithms based on convolutional neural network (CNN) provide iterative algorithms [15] in a coarse-to-fine manner to relieve the interference of complex background. Roth et al. first proposed a probabilistic bottom-up, coarse-to-fine approach for pancreas segmentation [16] where a multilevel deep ConvNet model is utilized to learn robust pancreas features. Two subsequent holistically nested segmentation networks [17, 18] advanced this previous work [16]. Zhou et al. presented a two-stage, fixed-point approach for the pancreas segmentation, which utilized the predicted segmentations from coarse model to localize and obtain smaller pancreas regions, which were further refined by another model [14]. Yu et al. presented the recurrent saliency transformation network to tackle the challenge of small organ segmentation where a saliency transformation module is utilized to connect coarse and fine stage to realize joint optimization [19]. Cai et al. designed a convolutional neural network equipped with convolutional LSTM to impose spatial contextual consistency constraints on successive image slices [20]. Cai et al. [21] further improved the pancreas initial segmentation in [20] by aggregating the multiscale, low-level features and strengthened the pancreatic shape continuity by bidirection recurrent neural network (BiRNN). Liu et al. [22] used superpixel-based approach to obtain coarse pancreas segmentations, which were then used to train five same-architecture fully convolutional networks (FCNs) with different loss functions to achieve accurate pancreas segmentations. This method is evaluated on 82 public CT volumes and achieved a Dice coefficient of 84.10 ± 4.91%. Man et al. [23] proposed a two-stage method composed of deep *Q* network (DQN) and deformable U-Net for the pancreas segmentation, in which DQN is used to obtain context-adaptive, coarse pancreas segmentations, which were then input to deformable U-Net for refinement. Zhu et al. [24] proposed a 3D coarse-to-fine network to segment the pancreas. This 3D method outperformed the 2D counterpart due to the full usage of the rich spatial information along the long axial dimension. Some common techniques such as dense connection [25], residual block, and sparse convolution [26, 27] are also widely utilized to segment the pancreas.

Google DeepMind proposed a spatial transformer [28], which is the first work to allow neural networks learn the transformation matrix from data and transform feature maps spatially. Specifically, spatial transformer network (STN) can globally deform feature maps through learned transformations, such as scaling, cropping, rotation as well as nonrigid deformation. Recently, Dai et al. proposed a deformable convolution to get over the limitation of fixed receptive field in standard convolution [29]. In detail, convolutional kernel with explicit offsets learned from the previous feature maps can adaptively change predefined receptive field in order to extract more target features. The specific deformable convolution is shown in Figure 2, in which some standard convolution layers are first utilized to learn and regress the deformation displacements for each sampling point in the image, and then the learned displacements are added to original sampling positions of the 2D convolution to enable network extract relevant and rich features far from original fixed neighborhood [30]. Different from STN [28], deformable convolution adopts a local and dense, instead of global manner to warp feature maps. Moreover, deformable convolution focuses on learning explicit offset for each neuron instead of kernel weights. Since the pancreas has various scales and shapes across patients and traditional convolutional kernel cannot address well on organs with high deformation due to the fixed receptive field, we believe deformable convolution is more suitable for the task of pancreas segmentation [31].

In this paper, we propose a semiautomated deformable U-Net model utilizing the power of U-Net and Deformable-ConvNets. The proposed architecture for pancreas segmentation has two merits. First, deep segmentation networks such as FCN [9], U-Net [10], and DeepLab [32] easily suffer from confusion by the large, irrelevant background information due to the small size of the pancreas in the entire abdominal CT volume. Motivated by [14], we take a similar strategy, i.e., first manually shrink the size of input image and then refine the extracted pancreas regions by the proposed deformable U-Net. The proposed method has the capability to extract the geometry-aware features of the pancreas with the help of deformable convolution. Second, we propose a novel loss function, focal generalized Dice loss (FGDL) function, to balance the size of foreground and background and enhance the ability of network for small organ segmentation. A conference version of this work was published in ISICDM 2019 [33]. In this extended version, we provide a more comprehensive description of literature review and detailed analysis of the proposed method and experimental investigation. The main modifications include presenting and analyzing the difference between standard convolution block and deformable convolution block (as shown in Figure 3), adding and analyzing the visualization results of the proposed DUNet (as shown in Figures 4 and 5), as well as the comparison results between the proposed DUNet and two baseline methods on the NIH dataset [34] (as shown in Figure 6 and Table 1), adding more evaluation metrics for testing the performance of the proposed DUNet (as shown in (9)–(11)), conducting new experiment to demonstrate the effectiveness of the proposed loss function for pancreas segmentation (as shown in Table 2), discussing advantages and limitations of the proposed DUNet, and adding more references.

## 2. Materials and Methods

In this section, a semiautomated deformable U-Net is proposed to segment the pancreas. Our method is built upon U-Net, which employed skip connections to aggregate multiple feature maps with the same resolution from different levels to recover the grained details lost in decoder branch and thus strengthen the representative capability of network. Since the pancreas only occupies a small fraction of the whole scan and the large and complex background information tends to interfere or confuse semantic segmentation framework, such as U-Net [10], we followed cascade-based methods [5, 12, 14], i.e., first localize target regions and then refine the extracted regions. Specifically, we first estimate the maximum and minimum coordinates of the pancreas to approximately locate its and then input the extracted pancreas regions to the refinement segmentation model to improve segmentation accuracy. Here, we designed a deformable U-Net (abbreviated as DUNet), as the refinement model. The key component in DUNet is deformable convolution, which can adaptively augment the sampling grid by learning 2D offsets from each image pixel according to the preceding feature maps. Incorporating deformable convolution into the baseline U-Net can improve the geometry-aware capability of U-Net. The overall structure of the proposed method is shown in Figure 7.

### 2.1. Network Architecture

Our approach is an encoder-decoder structure, designed for pancreas segmentation. As shown in Figures 7 and 3, the proposed architecture includes the standard convolution block, deformable convolution block, skip connection, downsampling, and upsampling. Considering that the deformable convolution block requires a little more computing resources and the aim of deformable convolution block is to help the network capture low-level, discriminative details at various shapes and scales, in order to balance the efficiency and accuracy, we experimentally apply the deformable convolution in the second and third layers of U-Net. Specifically, we replaced the standard convolution block of the second and third layers in the encoder, as well as the counterpart layers in the decoder with deformable convolution block.  Figure 3(b) shows the component of deformable convolution block. Concretely, each deformable convolution block is composed of convolutional offset layer, followed by convolution layer, BN [35], and ReLU layer, in which convolutional offset layer plays an important role in telling U-Net how to deform and sample feature maps [36]. The advantage of deformable convolution block is to utilize changeable receptive fields to effectively learn pancreas features with various shapes and scales.

Here, we describe the standard convolution and deformable convolution in detail. On the one hand, the standard 2D convolution can be seen as the weighed sum over a regular 2D sampling grid with weight *W*. For the 3 × 3 sized kernel with the dilation value of 1 (as shown in Figure 8(a)), the sampling grid *𝒢* in standard convolution defines the receptive field size and can be given by

(1) $$\begin{array}{c} G=\left\{\left(-1,-1\right),\left(-1,0\right),\ldots ,\left(0,1\right),\left(1,1\right)\right\}. \end{array}$$

The value of each location *p*_0_ on the output feature map *Y* can be calculated as

(2) $$\begin{array}{c} Y\left(p_{0}\right)=\sum_{p_{n}\in G}W\left(p_{n}\right)\cdot X\left(p_{0}+p_{n}\right), \end{array}$$

where *p*_*n*_ enumerates all locations in 2D sampling grid *𝒢*. On the other hand, rather than using the predefined sampling grid, deformable convolution automatically learns offset △*p*_*n*_ to augment the regular sampling grid and is calculated as

(3) $$\begin{array}{c} Y\left(p_{0}\right)=\sum_{p_{n}\in G}W\left(p_{n}\right)\cdot X\left(p_{0}+p_{n}+△p_{n}\right). \end{array}$$

In particular, the 2D deformable convolution can be mathematically formalized as follows:

(4) $$\begin{array}{c} \left(W^{{}^{\circ}}X\right)\left(i,j\right)=\sum_{m=-1}^{1}\sum_{n=-1}^{1}W\left(i,j\right)\times X\left(i-m+\delta_{i,j,m,n}^{\text{verticle}},j-n+\delta_{i,j,m,n}^{\text{horizontal}}\right),\;\forall i=1,\ldots ,H,\;\forall j=1,\ldots ,N, \end{array}$$

where ° denotes the deformable convolution operation, *W* is a 3 × 3 kernel with pad 1 and stride 1, *X* is the image with height *H* and width *N*, and (*i*, *j*) denotes the location of pixel in image. *δ*_*i*,*j*,*m*,*n*_^verticle^ and *δ*_*i*,*j*,*m*,*n*_^horizontal^ denote the vertical offset and the horizontal offset, respectively, which are learned by additional convolution on the preceding feature maps. Since the learned offset is usually not an integer, we performed bilinear interpolation on the output of the deformable convolutional layers to enable gradient back-propagation available.

### 2.2. Loss Function

Since the pancreas occupies a small region relative to the large background and Dice loss is relatively insensitive to class-imbalanced problem, most pancreas segmentation works adopt soft, binary Dice loss to optimize pancreas segmentation, and it is defined as follows:

(5) $$\begin{array}{c} L\left(P,G\right)=1-\frac{\sum_{i=1}^{N}p_{i}g_{i}+\varepsilon }{\sum_{i=1}^{N}p_{i}+g_{i}+\varepsilon }-\frac{\sum_{i=1}^{N}\left(1-p_{i}\right)\left(1-g_{i}\right)+\varepsilon }{\sum_{i=1}^{N}\left(2-p_{i}-g_{i}\right)+\varepsilon }, \end{array}$$

where *g*_*i*_ ∈ {0,1} and *p*_*i*_ ∈ [0,1] correspond to the probability value of a voxel in the manual annotation *G* and the network prediction P, respectively. *N* and *ϵ* denote the total number of voxels in the image and numerical factor for stable training, respectively. However, Dice loss does not consider the impact of region size on Dice score. To balance the voxel frequency between the foreground and background, Sudre et al. [37] proposed the generalized Dice loss, which is defined as follows:

(6) $$\begin{array}{c} \text{GDL}=1-2\frac{\sum_{l=1}^{2}w_{l}\sum_{i}^{N}p_{li}g_{li}}{\sum_{l=1}^{2}w_{l}\sum_{i}^{N}p_{li}+g_{li}}, \end{array}$$

where coefficient *w*_*l*_=1/(∑_*i*=1_^*N*^*g*_*li*_) is a weight for balancing the size of region.

Pancreas boundary plays an important role in dealineating the shape of pancreas. However, the pixels around the boundaries of the pancreas are hard samples, which are difficult to delineate due to the ambiguous contrast with the surrounding tissues and organs. Inspired by the focal loss [38, 39], we propose a new loss function, the focal generalized Dice loss (FGDL) function, to alleviate class-imbalanced problem in the pancreas segmentation and allow network to concentrate the learning on those hard samples, such as boundary pixels. The focal generalized Dice loss function can be defined as follows:

(7) $$\begin{array}{c} \text{FGDL}=\sum_{l=1}^{2}{\left(1-2\frac{w_{l}\sum_{i}^{N}p_{li}g_{li}+\varepsilon }{w_{l}\sum_{i}^{N}p_{li}+g_{li}+\varepsilon }\right)}^{1/\gamma }, \end{array}$$

where *γ* varies in the range [1, 3]. We experimentally set *γ*=4/3 during training.

## 3. Experiments

### 3.1. Dataset and Evaluation

We validated the performance of our algorithm on 82 abdominal contrast-enhanced CT images which come from the NIH pancreas segmentation dataset [34]. The original size of each CT scan is 512 × 512 with the number of slices from 181 to 460, as well as the slice thickness from 0.5 mm to 1.0 mm. The image intensity of each scan is truncated to [−100,240] HU to filter out the irrelevant details and further normalized to [0,1]. In this study, we cropped each slice to [192,256]. For fair comparisons, we trained and evaluated the proposed model with 4-fold cross validation.

Four metrics including the Dice Similarity Coefficient (DSC), Precision, Recall, and F-measure (abbreviated as *F*_1_) [40] are used to quantitatively evaluate the performance of different methods.

(1) Dice Similarity Coefficient (DSC) measures the volumetric overlap ratio between the ground truths and network predictions. It is defined as follows [41]:
  (8) $$\begin{array}{c} \text{DSC}=\frac{2\left\|V_{gt}\cap V_{\text{seg}}\right\|}{\left\|V_{gt}\right\|+\left\|V_{\text{seg}}\right\|}. \end{array}$$
(2) Precision measures the proportion of truly positive voxels in the predictions. It is defined as follows:
  (9) $$\begin{array}{c} \text{Precision}=\frac{\left\|V_{gt}\cap V_{\text{seg}}\right\|}{\left\|V_{\text{seg}}\right\|}. \end{array}$$
(3) Recall measures the proportion of positives that are correctly identified. It is defined as follows:
  (10) $$\begin{array}{c} \text{Recall}=\frac{\left\|V_{gt}\cap V_{seg}\right\|}{\left\|V_{seg}\right\|}. \end{array}$$
(4) *F*-measure shows the similarity and diversity of testing data. It is defined as follows:

(11) $$\begin{array}{c} F‐\text{measure}=2\cdot \frac{\text{Precision}\cdot \text{Recall}}{\text{Precision}+\text{Recall}}, \end{array}$$

where *V*_*gt*_ and *V*_seg_ represent the voxel sets of manual annotations and network predictions, respectively. For DSC, the experimental results are all reported as the mean with standard deviation over all 82 samples. For Precision, Recall, and F-measure metrics, we just reported the mean score over all 82 samples.

### 3.2. Implementation Details

The proposed method was implemented on the Keras and TensorFlow platforms and trained using Adam optimizers for 10 epochs on a NVIDIA Tesla P40 with 24 GB GPU. The learning rate and batch size were set to 0.0001 and 6 for training, respectively. In total, the trainable parameters in the proposed DUNet are 6.44 M, and the average inference time of our DUNet per volume is 0.143 seconds.

### 3.3. Qualitative and Quantitative Segmentation Results

To assess the effectiveness of deformable convolution in the pancreas segmentation, we compared the three models: Deformable-ConvNet, U-Net, and DUNet. To make the output size of Deformable-ConvNet to be the same as input, we make modification on Deformable-ConvNet [29] by substituting the original fully connected layers with upsampling layers. Figure 6 qualitatively shows the improvements brought by deformable convolution. It can be observed that our DUNet focuses more on the details of the pancreas, which demonstrates that deformable convolution can extract more pancreas information and enhance the geometric recognition capability of U-Net.

The quantitative comparisons of different models in terms of the Precision, Recall, *F*_1_, and mean DSC are reported in Table 1. It can be observed that our DUNet outperforms the modified Deformable-ConvNet and U-Net with improvements of average DSC up to 5.22% and 0.55%. Furthermore, it is worth noting that our proposed DUNet reported the highest average F-measure with 88.78%, which demonstrates that the proposed DUNet is a high-quality segmentation model and more robust than other two approaches. Figures 4 and 5 visualize the 2D and 3D overlap of segmentations from the proposed DUNet with respect to the manual segmentations, respectively. Visual inspection of the overlapping maps shows that the proposed DUNet can fit the manual segmentations well, which further demonstrates the effectiveness of our method.

### 3.4. Impact of Loss Function

To assess the effectiveness of the proposed loss function, we test standard Dice loss and the proposed loss with DUNet, i.e., Dice loss and the proposed focal generalized Dice loss (FGDL); the segmentation performance of the DUNet with different loss function is reported in Table 2. It can be noted that DUNet with the proposed FGDL improves mean DSC by 0.96% and min DSC by 8.38% compared with Dice loss.

### 3.5. Comparison with Other Methods

We compared the segmentation performance of the proposed DUNet with seven approaches [14, 16, 17, 21–24] on the NIH dataset [34]. Note that the experimental results of other seven methods were obtained directly from their corresponding literatures. As shown in Table 3, our method achieves the min DSC of 77.03%, max DSC of 93.29%, and mean DSC of 87.25 ± 3.27%, which outperforms all comparison methods. Moreover, the proposed DUNet performed the best in terms of both standard deviation and the worst case, which further demonstrates the reliability of our method in clinical applications.

## 4. Discussion

The pancreas is a very important organ in the body, which plays a crucial role in the decomposition and absorption of blood sugar and many nutrients. To handle the challenges of large shape variations and fuzzy boundaries in the pancreas segmentation, we propose a semiautomated DUNet to adaptively learn the intrinsic shape transformations of the pancreas. In fact, DUNet is an extension of U-Net by substituting the standard convolution block of the second and third layers in the encoder and counterpart layers in the decoder of U-Net with deformable convolution. The main advantage of the proposed DUNet is that DUNet utilizes the changeable receptive fields to automatically learn the inherent shape variations of the pancreas, then extract robust features, and thus improve the accuracy of pancreas segmentation.

There are several limitations in this work. First, during data processing, we first need radiologists to approximately annotate the minimum and maximum coordinates of the pancreas in each slice in order to localize it and thus reduce the interference brought by complex background. This work may be laborious. Second, the trainable parameters are relatively excessive. In future work, we will further improve pancreas segmentation performance from two aspects. First, we will explore and adopt attention mechanism to eliminate localization module and construct a lightweight network. Second, we will consider how to fuse prior knowledge (e.g., shape constraint) to the network.

## 5. Conclusions

In this paper, we proposed a semiautomated DUNet to segment the pancreas, especially for the challenging cases with large shape variation. Specifically, the deformable convolution and U-Net structure are integrated to adaptively capture meaningful and discriminative features. Then, a nonlinear Dice-based loss function is introduced to supervise the DUNet training and enhance the representative capability of DUNet. Experimental results on the NIH dataset show that the proposed DUNet outperforms all the comparison methods.

## Figures and Tables

**Figure 1:** Examples of 2D CT slices with pancreas annotations (red regions), showing the highly variable shape and size of pancreas. The largest area of pancreas is less than 0.8% of entire slice while the smallest area is less than 0.1% (best viewed in color).

**Figure 2:** Illustration of 3 × 3 deformable convolution. Offset field is generated from the preceding feature maps, and the number of output channels is 2*N*.

**Figure 3:** The comparison between (a) standard convolution block and (b) deformable convolution block.

**Figure 4:** Comparisons of 2D pancreas segmentations from the proposed DUNet with the manual segmentations. The first, second, and third columns denote the CT slices with their segmentations and bounding boxes of pancreas (red), the manual segmentations, and the network predictions, respectively. The last column denotes the overlapped maps between the network predictions and manual segmentations, with overlapped regions marked by magenta. (a) Original. (b) Groundtruth. (c) Prediction. (d) Overlapped.

**Figure 5:** Comparisons of 3D pancreas segmentations from the proposed DUNet with the manual segmentations. The first, second, and third columns denote the manual segmentations, the network predictions, and the overlapped maps between the network predictions and manual segmentations, respectively. The manual segmentations are shown in red, and the network predictions are shown in light green. (a) Label. (b) Prediction. (c) Overlapped.

**Figure 6:** Comparison of segmentation results between different models on the NIH dataset. (a) Original images with their segmentations and bounding boxes of pancreas (red). (b) The ground truths. (c–e) The predictions generated by our DUNet, U-Net, and Deformable-ConvNet, respectively.

**Figure 7:** An overview of the proposed DUNet. Input data are progressively convolved and downsampled or upsampled by factor of 2 at each scale in both encoding and decoding branches. Schematic of the standard convolution block and deformable convolution block is shown in Figure 3.

**Figure 8:** Comparisons of the sampling points in 3 × 3 standard and deformable convolution. (a) Sampling points (marked as blue) of standard convolution. (b) Deformed sampling points (marked as red) with learned displacements (pink arrows) in deformable convolution. (c-d) Two cases of (b), illustrating that the learned displacements contain translation and rotation transformations.

**Table 1:** Quantitative comparisons between the three different models on the NIH dataset. Bold denotes the best.

Model	F-measure	Recall	Precision	Mean DSC
Modified Deformable-ConvNet	0.8201	0.8084	0.8378	0.8203
U-Net	0.8738	**0.9010**	0.8499	0.8670
DUNet(Ours)	**0.8878**	0.8997	**0.8898**	**0.8725**

**Table 2:** Comparison of the DUNet with Dice loss (DL) and the proposed loss (DSC%). Bold denotes the best.

Method	Min DSC	Max DSC	Mean DSC
DUNet + DL	68.65	93.18	86.29 ± 4.33
DUNet + FGDL(Ours)	**77.03**	**93.29**	**87.25 ± 3.27**

**Table 3:** Comparison with other segmentation methods on the NIH dataset (DSC%). Bold denotes the best.

Method	Min DSC	Max DSC	Mean DSC
Roth et al., MICCAI'2015 [16]	23.99	86.29	71.42 ± 10.11
Roth et al., MICCAI'2016 [17]	34.11	88.65	78.01 ± 8.20
Zhou et al., MICCAI'2017 [14]	62.43	90.85	82.37 ± 5.68
Cai et al., 2019 [21]	59.00	91.00	83.70 ± 5.10
Liu et al., IEEE access 2019 [22]	N/A	N/A	84.10 ± 4.91
Zhu et al., 3DV'2018 [24]	69.62	91.45	84.59 ± 4.86
Man et al., IEEE T MED IMAGING 2019 [23]	74.32	91.34	86.93 ± 4.92
DUNet(Ours)	**77.03**	**93.29**	**87.25 ± 3.27**

## Data Availability

Pancreas CT images used in this paper were from a public available pancreas CT dataset, which can be obtained from http://doi.org/10.7937/K9/TCIA.2016.tNB1kqBU.
